The article "Effectiveness of Physical Activity and Finger Millet-Based Food Supplement on Biochemical Parameters and Bone Mineral Density among Premenopausal Women" was published in 2021. Journal: Evid Based Complement Alternat Med.

# Effectiveness of Physical Activity and Finger Millet-Based Food Supplement on Biochemical Parameters and Bone Mineral Density among Premenopausal Women

**DOI:** 10.1155/2021/4757991

**Published:** 2021-10-18

**Authors:** Golda Sahaya Rani, Aruna Swaminathan, Rajagopalan Vijayaraghavan

**Affiliations:** ^1^Sri Sathya Sai College of Nursing, Chengalpet 603108, India; ^2^Department of Nursing, Jazan University, Jazan, Saudi Arabia; ^3^Department of Research and Development, Saveetha Institute of Medical and Technical Sciences, Chennai 602105, India

## Abstract

The effectiveness of physical activity and finger millet-based food supplement on biochemical parameters and bone mineral density (BMD) among premenopausal women were studied. Serum calcium, phosphorus, alkaline phosphatase, and BMD of 720 women (30–40 years) were analyzed. From them, 150 women with low BMD (*t*-score, −1 to −2.5) and low calcium (<9.0 mg/dL) were randomized to control and experimental groups, equally. The experimental group was given 5 days per week physical activity, for 3 months, and a diet supplement of finger millet-based sweet balls (ragi laddu), 3 days per week for 3 months. The above parameters were measured as the posttest. Physical activity was assessed by the General Practice Physical Activity Questionnaire. A 24 h recall assessment was carried out for the diet supplement, and self-reported activity checklist was maintained for physical activity. Among 720 women, 163 (22.6%) showed BMD, *t*-score < −1.0, and calcium <9.0 mg/dL (*p* < 0.001). The serum phosphorus and alkaline phosphatase were also low (*p* < 0.001). After the supplementation to the experimental group, all the biochemical parameters, BMD, and physical activity score showed significant improvement in the posttest (*p* < 0.001). This study showed significantly low BMD and calcium among premenopausal women. Physical activity and finger millet supplement improved the calcium level and BMD.

## 1. Introduction

Osteoporosis is a global public health problem leading to increased bone fracture [1]. A study in Indian women showed 36% with osteopenia and 4% with osteoporosis. Low bone mineral density (BMD) was reported with the advancement of age and the menopausal status [2]. The high incidence of low bone density in women is due to decreased estrogen production during menopause [3]. There is calcium deficiency and a reduction in BMD. Women should have routine bone test and effective care to prevent complications [4]. Fractures caused by osteoporosis are important public health concern. Low BMD is common in women over the age of 40 and particularly after menopause [5].

To prevent osteopenia and osteoporosis, calcium and vitamin D supplements are required. Food containing high calcium, potassium, magnesium with vitamins and other minerals, viz., phosphorus, iron, and zinc are preferable for the normal bone metabolism to control osteopenia and osteoporosis [6]. Nutrition is an essential factor in maintaining the bone mass, particularly vegetable consumption [7]. Several millet grains also have a very high nutritive value, and among them, finger millet (*Eleusine coracana*, ragi in Hindi) is rich in calcium, protein, and essential amino acids [8]. Finger millet grain is popular in Asian and African countries due to the health benefits [9, 10]. Finger millet is considered as a super cereal in the United States. In more than 25 countries across Africa and Asia, finger millet is used accounting for 12% of the total millet consumption. Finger millet is used in cakes, pudding, and porridge [11]. Finger millet provides amino acid methionine, which is deficient in other starch cereals. Millets are gluten-free and processed as millet flour for use. It is a rich source of phosphorus, iron, magnesium, calcium, and fiber [12]. Finger millet has 5–30 times more calcium than other grains [13].

The article "Effectiveness of Physical Activity and Finger Millet-Based Food Supplement on Biochemical Parameters and Bone Mineral Density among Premenopausal Women" was published in 2021. Journal: Evid Based Complement Alternat Med.

Physical activity is essential for bone gain, and activities such as weight-bearing activities and muscle strengthening are recommended for a healthy bone [14, 15]. Physical activity has been shown to improve balance, bone growth, range of motion, and preserve bone mass. Regular physical activity in the early life strengthens the hip and prevents osteoporosis [16, 17]. Hence, it is important to create awareness to prevent bone deterioration from the premenopausal period [18].

Healthcare professionals should be aware of bone loss in various disease conditions and should prevent it with proper intervention supported by clinical biomarkers [19]. Osteoporosis prevention initiatives for premenopausal women are required for bone health and avoid bone loss. Several methods are available to prevent bone loss. In the present study, the effectiveness of physical activity and finger millet-based food supplement was evaluated on biochemical parameters and BMD among premenopausal women.

## 2. Materials and Methods

### 2.1. Participants

720 women of premenopausal age (30–40 years), members of a private women's organization (Kanchi Women's Sangamam Mutual's, Tamil Nadu, India), were initially screened for BMD and biochemical parameters. Among them, 150 women with BMD, *t*-score of −1 to −2.5, and serum calcium <9.0 mg/dL were included in this study. They were divided into control and experimental groups, equally by a random number table. Women with mental health problem and other systemic disease were excluded from the study. This study was approved by Institutional Ethics Committee of Saveetha Medical College and Hospital, Chennai (SMCH-IEC/006/04/2019), and carried out between May 2019 to April 2020. An information sheet was provided in English and local language (Tamil) to each participant, and signed consent to participate in the study was obtained.

The article "Effectiveness of Physical Activity and Finger Millet-Based Food Supplement on Biochemical Parameters and Bone Mineral Density among Premenopausal Women" was published in 2021. Journal: Evid Based Complement Alternat Med.

### 2.2. Methodology

Serum calcium (Ca), phosphorus (P), and alkaline phosphatase (ALP) were analyzed by an autoanalyzer as per manufacture's procedure (Microlab 300, ELITechGroup, France), and BMD was measured by an ultrasound bone densitometer (CM-200, Furuno Electric Co., Ltd., Japan) for all the 720 women. The 557 premenopausal women who did not meet the criteria (BMD, *t*-score of −1 to −2.5 and serum calcium <9.0 mg/dL) were excluded, and 13 women who did not volunteer to the osteoporosis prevention program due to personal reasons were also excluded. The 150 women who gave the signed consent for the intervention study were allocated randomly to the control and experimental groups. Pretest information on demographic profile by the questionnaire was recorded. The osteoporosis prevention program for the experimental group consisted of general awareness, physical activity, and diet supplementation. Structured education was provided once, on osteoporosis prevention (flash cards for 20 min). The physical activity consisted of spine (resistance), hip (strengthening), shoulder (resistance), and knee (strengthening). Pamphlets were given to the experimental group women after demonstration and was instructed to continue for 5 days a week for 3 months. Ragi laddu (finger millet sweet ball) supplement was given to the experimental group, three days per week for 3 months. The laddu was prepared using ragi flour (800 g), powdered jaggery (400 g), and ghee (300 g). 100 g of ghee was heated in a frying pan and ragi was roasted for 5 min in low flame. Powdered jaggery was added slowly and remaining ghee was poured, and mixed thoroughly. After cooling, the mixture was divided into 10 equal parts and made into laddu (150 g). All hygienic precautions were adhered in the preparation of the laddu by one of the investigators. The laddu was prepared every week fresh and 3 pieces were distributed to each experimental group women during the weekly meeting. A 24 h recall assessment was carried out for the diet supplement, and self-reported activity check list was maintained physical activity. The prepared laddu was certified by an approved food testing laboratory (Chennai Testing Laboratory Pvt. Ltd., India). At the end of the experimentation, analysis of serum calcium, phosphorus, and alkaline phosphatase and BMD were carried out for both control and experimental groups as the posttest.

The article "Effectiveness of Physical Activity and Finger Millet-Based Food Supplement on Biochemical Parameters and Bone Mineral Density among Premenopausal Women" was published in 2021. Journal: Evid Based Complement Alternat Med.

The physical activity was assessed by the General Practice Physical Activity Questionnaire (GPPAQ). For the assessment of physical activity, the General Practice of Physical Activity Questionnaire (GPPAQ) can be used which consists of seven self-explanatory questions and can be answered within one minute. The GPPAQ is a self-assessment physical activity questionnaire and is commonly used in primary care. The GPPAQ includes type of physical activity, duration, and walking speed and is designed for adults. A physical activity index can be computed and categorized as active, moderately active, moderately inactive, and inactive. [20, 21]. The levels of serum calcium, phosphorous, and alkaline phosphatase (ALP) were measured as biochemical indicators of bone turnover. ALP is a well-known marker for bone disorders [22].

### 2.3. Statistical Analysis

The data were analyzed by the *χ*^2^ test, Mann–Whitney rank sum test, Wilcoxon signed rank test, one-way ANOVA, and two-way repeated measures ANOVA with Bonferroni *t*-test for comparison of the variables. Linear regression was used for correlating the variables. Since the physical activity was assessed with a questionnaire, nonparametric statistics was used. For the biochemical and BMD measurements, parametric statistics was used assuming normal distribution. SigmaPlot 13 (Systat software, USA) was used for the statistical analysis and for plotting the graphs.

## 3. Results

Among the 720 women evaluated, 163 (22.6%) showed BMD less than −1.0 *t*-score with serum calcium less than 9.0 mg/dL (Table 1). *χ*^2^ analysis showed significant association with low BMD and low calcium level (*p* < 0.001). The serum phosphorus and ALP levels were also significantly low (*p* < 0.001), though there was no significant difference in the age (*p*=0.554).

Analysis of the laddu revealed 4.66 mg, 370 mg, and 133 mg of iron, calcium, and phosphorus, respectively, per 100 g. The protein content and fiber content were 4.0 g and 3.8 g per 100 g of laddu. The calculated energy was 372 kcal/100 g of laddu.

The control and experimental groups serum calcium, phosphorus, and ALP levels and BMD are shown in Figure 1. The mean ± SEM values of serum calcium of the control pretest, control posttest, experimental pretest, and experimental posttest were 6.95 ± 0.04, 6.94 ± 0.04, 7.04 ± 0.03, and 8.29 ± 0.02 mg/dL, respectively. Two-way RM ANOVA showed a significant difference among the groups (*p* < 0.001), pretest and posttest (*p* < 0.001), and the interaction (*p* < 0.001). There was no significant difference in the pretest (*p*=0.074), but the posttest showed a significant difference (*p* < 0.001) between control and experimental groups. The control pretest and posttest did not show a significant difference (*p*=0.446), while the experimental pretest and posttest showed a significant increase in the serum calcium level (*p* < 0.001). The mean ± SEM values of serum phosphorus of the control pretest, control posttest, experimental pretest, and experimental posttest are 1.86 ± 0.02, 1.84 ± 0.02, 1.84 ± 0.02, and 2.59 ± 0.02 mg/dL, respectively. Similar to serum calcium, serum phosphorus also showed a significant increase in experimental posttest only (*p* < 0.001). The ALP level of the control pretest, control posttest, experimental pretest, and experimental posttest was 29.9 ± 0.24, 29.7 ± 0.23, 29.2 ± 0.26, and 39.7 ± 0.30 U/L, respectively. Though the experimental posttest showed an elevated ALP level, it was within the clinical range.

The article "Effectiveness of Physical Activity and Finger Millet-Based Food Supplement on Biochemical Parameters and Bone Mineral Density among Premenopausal Women" was published in 2021. Journal: Evid Based Complement Alternat Med.

The mean ± SEM values of BMD of the control pretest, control posttest, experimental pretest, and experimental posttest are −1.80 ± 0.03, −1.80 ± 0.03, −1.73 ± 0.04, and −0.92 ± 0.04 g/cm^2^, respectively. Similar to serum calcium, there was significant improvement in the experimental posttest in BMD. There was no significant difference in the pretest (*p*=0.153), but the posttest (*p* < 0.001) showed a significant difference between control and experimental groups. The control pretest and posttest did not show a significant difference (*p*=0.928), while the experimental pretest and posttest showed a significant increase in BMD (*p* < 0.001).

Table 2 provides the effectiveness on physical activity in control and experimental groups, pretest and posttest. The experimental posttest showed significant improvement (*p* < 0.001) in the physical activity (from median of 0 to 3.2) compared to the control group (from median of 0 to 0) based on the GPPAQ.  Figure 2 shows the correlation of BMD with calcium, phosphorus, and ALP. A positive correlation was obtained among the variables showing the effectiveness of physical activity and the diet supplement in improving the BMD.

## 4. Discussion

Osteoporosis is not generally considered as a serious disease when compared to other communicable and noncommunicable diseases [23]. Nevertheless, osteoporosis-related fractures are highly associated with morbidity and mortality [24]. If properly diagnosed and preventive measures are adopted, the risk can be reduced to 50% [25]. Early diagnosis of osteopenia and osteoporosis in premenopausal women is required for a preventive management [26]. Deficiency in serum calcium was associated with osteopenia and osteoporosis [27]. In the present study 24.3% of premenopausal women showed low BMD and 51.7% showed low serum calcium. 22.6% showed low BMD as well as also low calcium in the premenopausal stage.

The article "Effectiveness of Physical Activity and Finger Millet-Based Food Supplement on Biochemical Parameters and Bone Mineral Density among Premenopausal Women" was published in 2021. Journal: Evid Based Complement Alternat Med.

Physical exercise has been shown to improve flexibility, strength, posture, and balance in women and also improve bone health [28]. Planned physical activity and sufficient intake of calcium are indicated for premenopausal women [27, 29]. Multicomponent exercise programme for 12 weeks was found to be suitable for improving the physical function and the quality of life for women with osteoporosis [30]. Weight-bearing and resistance exercises are the ideal lifestyle measures for prevention of osteoporosis among premenopausal women. The physical activity correlated with lowering the fat mass and increased BMD [31].

Several dairy products, vegetables, cereals, millets, and pulses are rich sources of calcium. Diet-based calcium supplement would be more acceptable and easier to practice [32]. Finger millet (ragi, *Eleusine coracana*) is a rich source of calcium and phosphorus and easily digestible [33]. It has been reported to have several beneficial effects, viz., blood glucose and cholesterol lowering, wound healing, and as a nutritional supplement for children also [34]. Finger millet has antioxidant and antibacterial properties [35]. Jaggery, also known as noncentrifugal sugar, is also rich in minerals and flavonoids [36]. In the present study, serum calcium was increased in the experimental posttest, as a result of the supplementation. Calcium increase is important for the bone metabolism. Dietary supplementation with calcium and vitamins D3 and B6 was found to be effective, improved the BMD, and increased calcium and ALP levels in the high fracture risk group who were undergoing medical rehabilitation [37]. In the present study also, it has been shown that an increase in serum calcium has improved the *t*-score of BMD, and a positive correlation was obtained with serum calcium and BMD (*r* = 0.761). Dairy products fortified with calcium and vitamin D to postmenopausal women has been shown to significantly influence BMD [38]. The daily requirement of calcium for Indian women is 600 mg [39]. 150 g of the finger millet laddu supplement would provide more than 500 mg of calcium and that has resulted in increased serum calcium, phosphorus, and BMD in the experimental posttest.

## 5. Conclusion

The present study shows significant low BMD and calcium among premenopausal women. Physical activity and finger millet supplement improved the calcium level and BMD. Women in the premenopausal stage should be aware of low BMD and its risk. They should improve their nutrition, particularly calcium from naturally available food products.

## Figures and Tables

**Figure 1:** Serum calcium, phosphorus, alkaline phosphatase, and bone mineral density in control and experimental groups of premenopausal women. Values are mean +SE (*n* = 75 each). Two-way RM ANOVA with the Bonferroni *t*-test. (a) Significantly different from the respective control group (between group). (b) Significantly different from the respective pretest (within group).

The article "Effectiveness of Physical Activity and Finger Millet-Based Food Supplement on Biochemical Parameters and Bone Mineral Density among Premenopausal Women" was published in 2021. Journal: Evid Based Complement Alternat Med.

**Figure 2:** Correlation of bone mineral density (BMD) with serum calcium (Ca), phosphorus (P), and alkaline phosphatase (ALP). Combined data of control and experimental posttest (*n* = 75 + 75).

**Table 1:** Classification of bone mineral density (BMD; *t*-score) and serum calcium (Ca, mg/dL) with serum phosphorus (P, mg/dL), alkaline phosphatase (ALP, U/L), and age (years) of premenopausal women.

S. No.	Category	BMD	Ca	Number	P	ALP	Age
1	Normal	>−1	<9.0	209	3.48 ± 0.57	82.5 ± 25.7	35.1 ± 3.1
			>9.0	336	3.48 ± 0.61	81.5 ± 26.3	34.8 ± 3.2
2	Osteopenia	−1 to −2.5	<9.0	153	1.97 ± 0.48^*∗*^	33.4 ± 15.1^*∗*^	34.8 ± 3.2
			>9.0	12	3.19 ± 0.55	87.3 ± 29.3	34.8 ± 3.1
3	Osteoporosis	<−2.5	<9.0	10	1.82 ± 0.16	30.0 ± 1.8	33.7 ± 3.2
			>9.0	0	-	-	-
Statistical analysis				*χ* ^2^ = 122.2 *P* < 0.001	*F* = 226.0 *P* < 0.001	*F* = 130.0 *P* < 0.001	*F* = 0.757 *P*=0.554

Values are mean ± SD (*n* = 720). *χ*^2^ analysis for BMD with Ca < 9.0 and >9.0 mg/dL groups. ^*∗*^Statistically significant from the respective Ca > 9.0 (mg/dL) group by one-way ANOVA with the Bonferroni *t*-test.

**Table 2:** Physical activity score of control and experimental groups of premenopausal women.

Groups	Mean	Median	Percentile	Statistical analysis			
				Between groups, Mann–Whitney rank sum test		Within groups, Wilcoxon signed rank test	
				Pretest Con/exp	Posttest Con/exp	Con Pre/post	Exp Pre/post
Con-pretest	0.047	0.0	0.0–0.0	*U* = 2779 *P*=0.781	*U* = 0 *P* < 0.001	*z* = 0.447 *P*=1.0	*z* = 7.550 *P* < 0.001
Con-posttest	0.048	0.0	0.0–0.0				
Exp-pretest	0.041	0.0	0.0–0.0				
Exp-posttest	3.165	3.2	3.0–3.4				

*n* = 75 each; Con, control; Exp, experimental.

## Data Availability

The data are available at the Department of Research and Development, Saveetha Institute of Medical and Technical Sciences, Chennai, India.
